# Clinical Observation of Alternative Wave Electroacupuncture Combined with Lee's Naprapathy in Treating Knee Osteoarthritis (Blood Stasis due to *Qi* Stagnation)

**DOI:** 10.1155/2022/2252551

**Published:** 2022-09-14

**Authors:** Hai-Jing Diao, Fei Li, Zi-Meng Lv, Hai-Ping Shi, Ya-Peng Nie, Zheng Gan, Ye-Fu Li, Guo-Rui Luan

**Affiliations:** ^1^Department of Tuina, The First Affiliated Hospital of Anhui University of Traditional Chinese Medicine, Hefei, Anhui 230601, China; ^2^The Third Ward, The Second Affiliated Hospital of Anhui University of Traditional Chinese Medicine, Hefei, Anhui 230061, China; ^3^Department of TuiNa, Anhui Integrated Traditional Chinese and Western Medicine Hospital, Hefei, Anhui 230031, China

## Abstract

**Objective:**

We aim to explore the clinical therapeutic effect of alternative wave electroacupuncture combined with Lee's naprapathy therapy on knee osteoarthritis (KOA) (blood stasis due to qi stagnation).

**Method:**

122 patients with KOA treated in our hospital from January 2018 to October 2021 were randomly grouped into a combined group (*n* = 61) and a control group (*n* = 61). The combined group was treated with alternative wave electroacupuncture combined with Lee's naprapathy, while the control group was treated with alternative wave electroacupuncture alone. Clinical efficacy of the two groups was observed. The Visual Analogue Scale (VAS), Lysholm Scale, Indexes of Severity for Osteoarthritis (ISOA), and Western Ontario and McMaster Universities Osteoarthritis Index (WOMAC) were compared before and after treatment, followed up for 3 months and 6 months. The adverse reactions of the two groups were observed.

**Result:**

The overall response rate of the combined group (96.72%) was higher than that of the control group (81.97%), and the difference was statistically significant (*P* < 0.05). After treatment and follow-up for 3 months and 6 months, the Lysholm score of the combined group was higher than that of the control group, while the VAS, ISOA, and WOMAC scores were lower than those of the control group, and the difference between the two was statistically significant (*P* < 0.05). There were no serious adverse reactions in both groups (*P* > 0.05).

**Conclusion:**

The alternative wave electroacupuncture combined with Lee's naprapathy is effective and safe in treating KOA (blood stasis due to *qi* stagnation).

## 1. Introduction

Knee osteoarthritis (KOA) is a bone and joint disease caused by degenerative changes in the articular and cartilage and subchondral bone and changes in joint mechanics, resulting in joint pain, deformity, and restricted movement. Clinically, it is a frequently occurring disease in middle-aged and elderly people [1, 2]. The main clinical manifestations of KOA include pain, swelling, and stiffness. In some severe cases, joint dysfunction and disability can be observed. It is an important reason for disability in the elderly and can seriously influence the quality of life of patients. Now, conservative treatment is mostly used in the early to mild-stage KOA. Traditional Chinese medicine (TCM) for KOA includes naprapathy and acupuncture. KOA is deemed as “bone paralysis” by TCM, a syndrome of deficiency in origin and excess in superficislity, and kidney deficiency and *qi* stagnation, as well as blood stasis, is the main mechanism of the disease. Previous studies reported that [3] electroacupuncture could effectively relieve pain and joint swelling in patients with osteoarthritis of the knee, unblocking the meridians, promoting circulation of *qi* and blood, promoting blood circulation and vasodilation, promoting the free radical release, improving the nutritional status of tendons and bones, regulating *qi* and blood nutrition, and repairing damaged cartilage tissue. Lee's naprapathy method is a type of technique that Professor Yefu Li has developed by combining the Hai School of Naprapathy and Xin'an medicine. We aim to investigate the efficiency of the combination of alternative wave electroacupuncture with Lee's naprapathy method in treating KOA with blood stasis due to qi stagnation.

## 2. Materials and Methods

### 2.1. Common Data

122 patients with KOA treated in our hospital from January 2018 to October 2021 were randomly divided into a combined group (*n* = 61) and a control group (*n* = 61). There were 25 males and 36 females in the combined group. The age ranged from 41 to 65 years with an average of (51.70 ± 6.18) years. The course of disease was 0.5∼4 years, with an average of (2.46 ± 0.95) years; Predilection sites: 33 cases of left knee joint, 28 cases of right knee joint. There were 27 males and 34 females in the control group. The age ranged from 40 to 68 years with an average of (52.00 ± 5.97) years. The course of disease was 0.5∼5 years, with an average of (2.58 ± 0.91) years; Predilection sites: 31 cases of left knee joint and 30 cases of right knee joint. The general data of the two groups were compared (*P* > 0.05), to find out which were comparable. This study was approved by the hospital ethics committee.

### 2.2. Western Medicine Diagnostic Criteria

The diagnosis was made according to the Diagnosis and Treatment Guide of Bone and Joint (2007) [4], ①Patient's age was 40 years or older; ②Patients' knee joints had been in pain and discomfort for 1 month; ③The time of morning stiffness was less than 3 min; ④X-ray examination showed degenerative changes of knee joint; ⑤There was fricatives in knee joint activities; ⑥The synovial fluid (at least twice) was clear and sticky, and the white blood cell count was less than 2000/ml. Those who meet ① + ② and ① + ③ + ⑤ + ⑥ requirements can be diagnosed as KOA.

### 2.3. TCM Diagnostic Criteria

According to the Consensus of TCM Diagnosis and Treatment Experts of Knee Osteoarthritis (2015) [5]. Syndrome differentiation standard of blood stasis due to *qi* stagnation: main symptom: joint tingling, aggravated after rest; Symptoms: dark complexion, dark-purple tongue or ecchymosis, sunken and astringent pulse.

### 2.4. Inclusive Criterion

①Patients meet the above diagnostic criteria of Chinese and Western medicine; ②Age ranged from 40 to 75 years; ③Patients did not take nonsteroidal anti-inflammatory drugs, immunosuppressants, and other drugs that affected the study one week before enrollment; ④Consent to conservative treatment; ⑤The patients volunteered to participate in this study.

### 2.5. Exclusive Criterion

①Patients with recent history of acute knee injury; ②Local skin damage and infection; ③Patients with knee joint tumor and rheumatoid arthritis; ④Patients with severe organ dysfunction such as heart, liver, and kidney; ⑤The knee joint function was severely deformed; ⑥Patients with consciousness dysfunction.

### 2.6. Method

The combined group was treated with alternative wave electroacupuncture combined with Lee's naprapathy, while the control group was treated with alternative wave electroacupuncture alone.

#### 2.6.1. Alternative Wave Electroacupuncture

Liangqiu point, Xuehai point, and internal and external knee eye points were positioned, the patient was placed in a supine position and the affected knee was disinfected. 0.30 mm × 40 mm disposable needles were used for the Xuehai point and Liangqiu point, and 0.3 mm × 75 mm disposable needles were used for the inner knee eye and Dubi point, the needle was stuck in at 30 mm and G6805-II electroacupuncture was used. Two groups of electroacupuncture were connected ipsilateral, one group was connected with Xuehai point and the inner knee eye point, and the other group was connected with Liangqiu and Dubi point. The frequency was set at 2 Hz/10 Hz, and the intensity was adjusted to make the patient feel soreness and swelling but could tolerate it, and the needles were left in place for 30 minutes.

#### 2.6.2. Lee's Naprapathy

The internal and external knee eyes point, Yanglingquan point, Xuehai point, Liangqiu point, Futu point, Zhizhong point, Chengshan point, and Fengshi point, etc. were included in acupuncture points, and the rolling, pressing and kneading, flicking, lifting, rubbing, and shaking were covered by naprapathy.

①Relaxation naprapathy: the patient was placed in a supine position and the rolling naprapathy was applied to the quadriceps muscle of the thigh, focusing on the upper patella, and the Xuehai point, Liangqiu point, Heding point, and Futu point were pressed for 1∼3 minutes each time. ②Adjustment naprapathy: pressing-lifting and flicking naprapathy were alternately applied to the patellar ligament and the medial and lateral collateral ligaments of the patients, focusing on the internal and external knee eye, Xuehai point, Liangqiu point, Yanglingquan point, and kneaded, and the patella was taken, 1∼3 minutes each time. The patient was placed in a supine position with the hip and knee flexed, the operator pressed the patella on the affected side with one hand, held the distal calf with the other hand and did a knee flexion and rocking naprapathy, together with knee rotation and flexion and extension for 1∼3 minutes each time. ③Ending naprapathy: rubbing naprapathy was applied around the affected knee until the patient felt the knee slightly warm, for 1 to 3 minutes each time. For painful swollen joints, rubbing the Yanglingquan point, Yinlingquan point, and Jiegu point could be used to relieve pain. Each treatment was repeated for 30 minutes, 3 times a week for 4 weeks.

### 2.7. Main Outcome Measures

①Clinical efficacy. ②VAS [6] was used to assess the pain of the two groups before and after treatment, and followed up for 3 and 6 months, the pain was rated from 0 to 10 according to the degree of pain. The higher scores represented the more severe the pain. ③Lysholm Scale [7] was used to assess the joint function of the two groups before and after treatment, and followed up for 3 and 6 months. According to the score, the joint function can be divided into poor (<50 points), fair (50∼74 points), good (75∼90 points), excellent (91∼99 points), and normal (100 points). ④ISOA [8] was used to evaluate the knee joint function of the two groups before and after treatment, and followed up for 3 and 6 months. The scale was divided into three dimensions: pain or discomfort, max, walking distance, and ADL. Each dimension scored 0–8 points, with a total score of 0–24 points. The higher the score, the worse the knee joint function. ⑤WOMAC [7] was used to assess the knee joint function of the two groups before and after treatment, and followed up for 3 and 6 months. The scale included three dimensions: pain (1∼5 items, 0∼20 points), stiffness (6∼7 items, 0∼8 points), and daily function (8∼24 items, 0∼68 points). Five-grade scoring method was used, and the score was from no difficulty to extreme difficulty. ⑥Comparison of adverse reactions between the two groups.

### 2.8. Assessment Standard of Therapeutic Effect

The therapeutic effects of the two groups were assessed according to the Assessment Standard of Orthopedic Diseases [9]. Clinical cure: knee joint function was recovered and symptoms disappeared; Markedly improvement: patients whose joint pain, swelling, and other symptoms are obviously relieved, joint function is obviously improved, or symptoms disappear completely, but relapse within one year and get better after treatment; Improvement: joint swelling and pain improved; Failure: clinical symptoms and signs are unchanged or aggravated.

### 2.9. Statistical Methods

SPSS 20.0 statistical software was used to analyze and process the data, and the measurement data were represented by *x*‾ ± *s*, *t*-test was used for comparison between the groups, and the paired *t*-test was used for comparison before and after treatment within groups. The counting data were expressed as frequency and composition ratio, and the *χ*^2^ test was used. The difference was statistically significant *P* < 0.05).

## 3. Results

### 3.1. Comparison of Clinical Efficacy

The overall response rate of the combination group (96.72%) was higher than that of the control group (81.97%), and the difference between the two was statistically significant (*P* < 0.05). See Table 1.

### 3.2. Comparison of VAS and Lysholm Scores

No statistically significant difference was found in VAS and Lysholm scores between the two groups before treatment (*P* > 0.05). The VAS scores decreased and Lysholm scores increased of the two after treatment and follow-up for 3 and 6 months. After treatment and follow-up for 3 and 6 months, the VAS scores of the combined group were lower than those of the control group, the Lysholm scores were higher than those of the control group, and the difference between the two was statistically significant (*P* < 0.05). See Table 2.

### 3.3. Comparison of ISOA Scores

No statistically significant difference was found in ISOA scores between the two groups before treatment (*P* > 0.05); pain or discomfort, maximum walking distance, and ADL scores of both groups decreased after treatment and were followed up for 3 and 6 months, . Pain or discomfort, maximum walking distance, and ADL scores of the combined group after treatment followed up for 3 and 6 months were lower than those of the control group, and the difference between the two was statistically significant (*P* < 0.05). See Table 3.

### 3.4. Comparison of WOMAC Scores

No statistically significant difference was found in WOMAC scores between the two groups before treatment (*P* > 0.05); The scores of arthrodynia, anchylosis, and joint function in the two groups decreased after treatment and were followed up for 3 and 6 months. The scores of joint pain, joint stiffness, and joint function in the combined group were lower than those in the control group, and the difference between the two was statistically significant (*P* < 0.05). See Table 4.

### 3.5. Comparison of Adverse Reactions

The patients of the two groups had no serious adverse reactions in the process of therapy.

## 4. Discussion

KOA belongs to the category of “bone paralysis” in TCM, the feature of the mechanism of the disease is that deficiency in origin and excess in superficislity, which is related to body tendons and veins losing nourishment, long-term strain, liver and kidney deficiency, exogenous cold, and damp evil. The liver governs the tendons, the kidney governs the bones, and tendons belong to bones and can constrain joints. The deficiency of the liver and kidneys in the middle-aged and elderly, kidney deficiency and marrow reduction, leading to tendons and bone loss are the root of this disease. The disease develops when phlegm and blood stasis intermingle and when wind, cold, and dampness attack. The kidneys are the main reservoir of the essence and the essence produces marrow and regenerates bone. The deficiency of kidney essence and the loss of nourishment of bone in middle-aged and elderly people manifest as atrophy and pain in the joints. Modern medical pathology has shown that the onset of knee osteoarthritis is influenced by genetic, environmental, and multiple biological factors [10–12]. Clinical treatments of osteoarthritis of the knee are mainly conservative and surgical. Surgical treatment can trigger negative emotions in patients and poor patient compliance, drug therapy and rehabilitation therapy are applied as the most commonly used conservative treatments. And drug treatment of nonsteroidal anti-inflammatory drugs can cause severe gastrointestinal reactions. In this study, alternative wave electroacupuncture combined with seven-step naprapathy was used for the treatment of KOA, in which electroacupuncture not only had an analgesic effect but also improved vascular spasm, reduced local edema and increased tissue excitability. Different wave types had different therapeutic effects, alternative waves can cause an inhibitory effect on motor nerves, with a good analgesic effect and lasting for a long time [13]. Previous studies [14–16] had shown that alternative waves could promote energy and metabolism, improved the flow of qi and blood, and had been widely used in the treatment of cervical spondylosis and other diseases [17, 18]. One of the main features of Chinese medicine was syndrome differentiation and treatment, and naprapathy was a common Chinese rehabilitation therapy. In the treatment of TCM naprapathy, many doctors emphasized the treatment of the disease but overlooked the grasp of the evidence. Li Yefu thought that naprapathy therapy should be in accordance with the way of thinking and followed the basic principle of “syndrome differentiation and treatment, take all the symptoms together,” and points were like drugs, different points had different functions. For example, acupuncture points such as Zusanli point, Qihai point, and Dazhi point can be used to circulate Qi, similar to the effects of Ginseng and Astragalus; acupuncture points such as Xuehai point and Sanyinjiao point could be used to circulate and invigorate blood, similar to the effects of Angelica Sinensis. According to the principle of “Monarch, minister, assistant and guide,” the appropriate naprapathy should be carried out regularly. The warm method was used for cold syndrome to relieve the exterior, and the purgation therapy was used for cold and sthenia syndrome to unclog. Compared with traditional naprapathy, Lee's naprapathy focused on the targeted massage of each acupuncture point during the process of naprapathy, and it could effectively improve local blood circulation and inflammatory response. Massaging the Yanglingquan point and other points could activate blood, clear collaterals, and eliminate the swelling. Results of the study showed that the total effective rate of the combined group (96.72%) was higher than that of the control group (81.97%), and the difference was statistically significant (*P* < 0.05). This indicated that alternative wave electroacupuncture with Lee's naprapathy was more effective in treating KOA. The flow of qi and blood was boosted by alternative wave electroacupuncture, and the blood circulation was improved by Lee's naprapathy.

In the study, the Lysholm scores of the combined group were higher than those of the control group, and the scores of VAS, ISOA, and WOMAC were lower than those of the control group before treatment, after treatment, and after 3 and 6 months of follow-up. The VAS was used to assess the patients' functional knee pain and the Lysholm, ISOA, and WOMAC were used to assess the patients' knee function. Data taken before and after treatment and at 3 and 6 months of follow-up in this study showed that alternative wave electroacupuncture with Lee's naprapathy is more effective in improving pain and knee function in patients with osteoarthritis of the knee, and the treatment is stable, with good treatment results maintained over the follow-up time. In this study, the acupuncture points selected for the electroacupuncture treatment were the inner knee eye belonging to extra nerve points and the Dubin point belonging to the stomach meridian of foot-Yangming, which were pressure points for osteoarthritis of the knee, and acupuncturing at these points can promote the release of endogenous morphine peptides to play an analgesic effect. Also, the Xuehai point was the main blood blockage, which can promote blood access through acupuncture, Liangqiu point was the point of qi accumulation, which can mediate qi and blood through acupuncture. Under the alternating wave, the inhibitory effect would occur in the sensory and motor nerves to achieve the good analgesic effect. Several previous studies had shown that alternative waves were more effective than continuous waves in improving pain in diseases [19, 20]. Correlational research had also shown that alternative waves could improve the flow of qi and blood, energy, and metabolism in the body, and alternative waves were better than continuous waves in improving joint pain and swelling [21, 22]. Lee's naprapathy was divided into the treatment into 3 parts: relaxation, adjustment, and ending. Firstly, relaxing the soft tissues, balancing muscle strength, relieving spasms and pain, promoting blood circulation, then making adjustments, which can correct the joints, and finally concluding the treatment with finishing techniques, which have the overall effect of restoring the elasticity of fibrous tissues, reducing interarticular pressure and promoting cartilage metabolism. Various naprapathy's step by step, in reasonable combination, can effectively improve pain and knee function. The inner and outer knee eye points and Heding point were included in extra nerve points. The inner knee eye was opposite to the outer knee eye, so naprapathy could open the channels and disperse cold, unblocking the joints. According to research, stimulating the inner and outer knee eyes could delay the pathological damage state of osteoarthritis, possibly by regulating the abnormally high serum levels of matrix metalloproteinase 1 and affecting the Wnt signaling pathway to slow down cartilage degeneration [23, 24]. Yanglingquan point was a point of the gallbladder meridian of foot-Shaoyang, which was the entry point of the spleen meridian and was the lower conjunction point of the lower confluent point of the gall bladder, which was responsible for the management of tendon injury disease, naprapathy can dredge joints. The Xuehai point and Liangqiu point are localized points in the knee joint. Naprapathy can regulate qi and open the meridians, reducing swelling and pain. The Wuizhong point was at the knee and could be used to improve joint movement and relieve pain. Futu point was included in the stomach meridian of foot-Yangming, Fengshi point was included in the gall bladder meridian and Chengshan point belongs to the bladder meridian, manipulating them has the effect of dispersing cold, detumescence, regulating qi and relieving pain, and if all points were manipulated, cold can be dispersed, the body's tendon and vessel could be unclogged and joints can be activated. The synergistic effect was formed by the action of the alternative wave electroacupuncture and Lee's naprapathy, knuckle pain, and knee joint function of patients were effectively improved by these two methods.

In conclusion, the alternative wave electroacupuncture combined with Lee's naprapathy method for the treatment of KOA had a significant effect on improving the pain and joint function of patients, and was safe and had clinical application value.

## Figures and Tables

**Table 1:** Comparison of clinical efficacy (cases (%)).

Groups	Clinical cure	Markedly improvement	Improvement	Failure	Total effectiveness
Combined (*n* = 61)	17 (27.87)	36 (59.02)	6 (9.84)	2 (3.28)	59 (96.72)
Control (*n* = 61)	10 (16.39)	25 (40.98)	15 (24.59)	11 (18.03)	50 (81.97)
*χ* ^*2*^ value					6.974
*P* value					0.008

**Table 2:** Comparison of VAS and Lysholm (*x* ± *s*, scores).

Groups	VAS				Lysholm			
	Before treatment	After treatment	3 M follow-up	6 M follow-up	Before treatment	After treatment	3 M follow-up	6 M follow-up
Combined (*n* = 61)	7.39 + 0.76	4.97 + 1.47^a^	1.67 + 0.98^a^	2.75 + 1.03^a^	59.13 + 5.35	77.28 + 6.70^a^	76.21 + 5.23^a^	74.77 + 6.29^a^
Control (*n* = 61)	7.31 + 0.92	5.70 + 1.09^a^	2.75 + 1.03^a^	4.34 + 1.05^a^	58.18 + 4.13	64.59 + 4.51^a^	69.89 + 4.97^a^	71.80 + 6.90^a^
*t*	0.536	3.151	6.180	8.467	1.098	12.262	6.847	2.482
*P*	0.593	0.002	<0.001	<0.001	0.274	<0.001	<0.001	0.014

*Note.* ^a^ *P* was <0.05 compared with that before treatment in the same group.

**Table 3:** Comparison of ISOA (*x* ± *s,* scores).

Groups	Pain or discomfort				Max. walking distance				ADL			
	Before treatment	After treatment	3 M follow-up	6 M follow-up	Before treatment	After treatment	3 M follow-up	6 M follow-up	Before treatment	After treatment	3 M follow-up	6 M follow-up
Combined (*n* = 61)	4.98 + 0.79	2.49 + 0.79^a^	2.38 + 0.58^a^	2.66 + 0.57^a^	4.82 + 0.85	2.77 + 0.64^a^	1.98 + 0.56^a^	2.36 + 0.68^a^	4.77 + 0.62	2.74 + 0.77^a^	2.10 + 0.72^a^	2.28 + 0.78^a^
Control (*n* = 61)	5.10 + 0.62	3.85 + 0.83^a^	3.02 + 0.65^a^	3.23 + 0.69^a^	4.84 + 0.66	3.10 + 0.81^a^	2.77 + 0.67^a^	3.21 + 0.82^a^	4.87 + 0.74	3.43 + 0.96^a^	2.87 + 0.78^a^	3.07 + 0.87^a^
*t*	0.893	9.266	5.746	4.981	0.119	2.476	7.037	6.240	0.797	4.373	5.638	5.257
*P*	0.373	<0.001	<0.001	<0.001	0.905	0.015	<0.001	<0.001	0.427	<0.001	<0.001	<0.001

*Note.* ^a^ *P* was <0.05 compared with that before treatment in the same group.

**Table 4:** Comparison of WOMAC (*x* ± *s,* scores).

Groups	Arthrodynia				Anchylosis				Joint function			
	Before treatment	After treatment	3 M follow-up	6 M follow-up	Before treatment	After treatment	3 M follow-up	6 M follow-up	Before treatment	After treatment	3 M follow-up	6 M follow-up
Combined (*n* = 61)	11.70 + 3.42	4.80 + 0.96^a^	2.72 + 1.36^a^	2.87 + 1.02^a^	5.61 + 0.90	2.64 + 0.98^a^	1.93 + 0.36^a^	1.89 + 1.02^a^	37.97 + 2.99	15.44 + 1.59^a^	12.00 + 2.88^a^	16.02 + 1.73^a^
Control (*n* = 61)	11.90 + 2.72	6.90 + 2.26^a^	6.21 + 1.25	6.56 + 1.88^a^	5.67 + 1.04	4.31 + 1.25^a^	3.39 + 1.31	3.62 + 1.13^a^	38.56 + 3.75	22.33 + 2.79^a^	19.38 + 4.44^a^	20.67 + 3.80^a^
*t*	0.352	6.663	14.772	13.481	0.372	8.228	8.405	8.932	0.961	16.776	10.881	8.707
*P*	0.726	<0.001	<0.001	<0.001	0.711	<0.001	<0.001	<0.001	0.338	<0.001	<0.001	<0.001

*Note.* ^a^ *P* was <0.05 compared with that before treatment in the same group.

## Data Availability

The labeled datasets used to support the findings of this study are available from the corresponding author upon request.
